# A Probabilistic Patient Scheduling Model with Time Variable Slots

**DOI:** 10.1155/2020/9727096

**Published:** 2020-09-01

**Authors:** Danae Carreras-García, David Delgado-Gómez, Enrique Baca-García, Antonio Artés-Rodriguez

**Affiliations:** ^1^Department of Statistics, Universidad Carlos III of Madrid, Universidad Carlos III de Madrid, Leganés, Spain; ^2^Department of Psychiatry, Fundación Jiménez Díaz Hospital, Madrid, Spain; ^3^Madrid Autonomous University, Madrid, Spain; ^4^Universidad Catolica del Maule, Talca, Chile; ^5^Signal Theory and Communications Department, Universidad Carlos III of Madrid, Leganés, Spain

## Abstract

One of the current challenges faced by health centers is to reduce the number of patients who do not attend their appointments. The existence of these patients causes the underutilization of the center's services, which reduces their income and extends patient's access time. In order to reduce these negative effects, several appointment scheduling systems have been developed. With the recent availability of electronic health records, patient scheduling systems that incorporate the patient's no-show prediction are being developed. However, the benefits of including a personalized individual variable time slot for each patient in those probabilistic systems have not been yet analyzed. In this article, we propose a scheduling system based on patients' no-show probabilities with variable time slots and a dynamic priority allocation scheme. The system is based on the solution of a mixed-integer programming model that aims at maximizing the expected profits of the clinic, accounting for first and follow-up visits. We validate our findings by performing an extensive simulation study based on real data and specific scheduling requirements provided by a Spanish hospital. The results suggest potential benefits with the implementation of the proposed allocation system with variable slot times. In particular, the proposed model increases the annual cumulated profit in more than 50% while decreasing the waiting list and waiting times by 30% and 50%, respectively, with respect to the actual appointment scheduling system.

## 1. Introduction

One of the current problems faced by health centers is the existence of patients who do not attend their appointments. These patients, commonly known as no-shows, cause damage which includes a drastic reduction in the health center's income and extend patients' access to medical care. No-show rates ranging from 4 to 79.2% [1] and losses reaching 150 million dollars only in the United States [2] have been reported.

In order to reduce these numbers, health centers use reminders and sanctions. However, several studies have shown that these strategies only achieve a slight or moderate reduction in the no-show rates [3, 4]. Moreover, it has been pointed out that sanctions may limit access to patients with limited income to medical centers [5], and automatic reminder systems might have an important economic impact on the health centers [6].

An alternative to these active strategies is the use of appointment scheduling systems. These systems aim at obtaining an allocation of the patients that reduce given performance measures, such us patient overtime or doctor idle time. The development of these patient scheduling systems is a very active field. Literature review articles covering seminal and more recent approaches include [7–9]. This vast productivity is a consequence of the large variety of peculiarities of the health centers that cause the systems to be practically tailor-made. In general terms, these systems can be differentiated according to (1) online vs. offline; (2) single vs. multiple servers; (3) appointment rules; (4) performance measures; (5) inclusion of environmental factors; and (6) modeling approach.

Regarding the first classification, systems can consider online **(**sequential) and offline (simultaneous) scheduling. Primary care centers usually assign the appointment at the time the patient requests it (online scheduling), while specialties assign it days later, after checking the doctors' availability and analyzing the required resources (offline scheduling) [10]. Online systems are more common in practice; however, they are more difficult to model. On the other hand, offline systems are becoming increasingly important as requests can be made automatically, and patients are notified later.

With respect to the second category, queuing theory allows the classification of these systems into single-server or multiple servers according to the number of providers being modelled at a time. The single-server assumption is usually associated with the fact that each doctor has their own set of patients associated. However, it is known that models based on multiple servers are more efficient, and in some cases, such as laboratories or x-rays tests, they are also optimal [7].

In terms of appointment rules, two parameters have to be considered. Firstly, the number of patients scheduled in each time slot (block-size), where the number of patients to be seen in the first slot (initial-block), is usually studied separately. Secondly, the time length of each slot (appointment interval) is being studied also. Each combination of these parameters describes an appointment rule. For example, individual-block/variable-interval describes the rule that assigns only one patient to each slot with variable time length.

Regarding performance measures, these are used to describe the objective pursued when creating a particular scheduling system. Most of the models are built from an optimization problem seeking to achieve the best allocation of patients; although, in some cases, heuristic rules are created that are then validated by simulation. These measures are usually associated with the cost of patient waiting time, or the doctor's idle time, the revenues of attending a patient, or a combination of them.

The inclusion of environmental factors into scheduling systems is still underdeveloped and a large consensus exists on it being one of the most promising lines to explore in future research. Cayirli and Veral [7] point out the importance of including no-shows, walk-in, urgent patient, emergencies, and second consultations in appointments scheduling systems. Although these factors can be addressed separately, through the center's policies, taking them into account can lead to better results. Gupta and Denton [8] add to these late cancellations, which are often classified along with no-shows, and patient preferences. More recently, Ahmadi et al. [9] add another environmental factor such as patient lack of punctuality, physician lateness, service interruption, random service time, and other patient appointment requirements.

As for the mathematical model used for the solution, most scheduling systems make use of stochastic optimization or dynamic stochastic programming scheduling, because these are more robust to random arrivals and random service times. However, the recent availability of Electronic Health Records (EHR) and advances in data science have made it possible to obtain more accurate predictions about these two factors, random arrivals and service times, making the use of deterministic planning systems possible. Most of the deterministic models are formulated using integer or mixed linear programming models aiming at optimizing some performance measure of the scheduling. This type of model is widely used in specialties, where deterministic service times and near-zero no-show probabilities are assumed [9].

In this paper, we propose a deterministic integer linear programming (ILP) model for offline scheduling of patients in the presence of heterogeneous no-shows and variable times services in a specialty service of a public health center. To the best of our knowledge, this is the first offline scheduling model that considers both heterogeneous patient no-shows and length variable appointment intervals. The system aims to maximize the expected revenues of the clinic considering the different show-rates of each patient during a whole week. The model is designed as a single-server given the fact that each doctor is assumed to have their own list of patients. The appointment rule used is individual-block/variable-interval, with no initial-block, for which only one patient is assigned to each variable time length slot.

In order to validate the model, experiments are carried out to reproduce the routine of the psychiatric department of the Fundación Jiménez Díaz Hospital in Madrid, Spain, for an entire year. In this sense, patient show rates are estimated, and three different appointment intervals with information provided by the center are incorporated into the proposed model. We also take into account other environmental factors such as large waiting lists, major revenues from scheduling new patients, and the dynamic priority assignment scheme. The performance of the model is compared with other scheduling systems, including the one proposed by Ruiz-Hernández et. al [11], which is currently implemented at the psychiatric department of this hospital, showing a considerable improvement.

The rest of the article is structured as follows. In Section 2, we present a literature review in scheduling systems in health centers with heterogeneous no-show probabilities. Next, in Section 2, the probabilistic patient scheduling problem with time-variable slots is introduced. In Section 3, the specific characteristics of scheduling in the health center basis for this study are described. In Section 5, the numerical experiments carried out to evaluate the model are presented and discussed. Finally, the article ends in Section 6 with the conclusions of the results obtained.

## 2. Literature Review

In this section, we review appointment scheduling systems that take into account variable appointment intervals and heterogeneous no-shows. First, we discuss models that consider different appointment intervals. Then, we move on to models with heterogeneous no-show probabilities. Finally, we will present the contributions of our proposal. A summary with the most recent works compared with the proposed method is presented in Table 1.

It is important to point out the difference between the appointment interval and the service time. The former is the scheduled length of an appointment, while the latter is the actual time the patient spends at the appointment. In works considering different appointment intervals, it is usually assumed that the service time is deterministic but unknown, so it can be estimated. Cayirli et al. [12] simulate different sequence and appointment rules on a variety of environmental factors, such as different service times for new and follow-up patients and the presence of homogeneous absences. Huang and Verduzco [13] reclassify patients into different types of visits and determine appointment length by incorporating performance measures such as patient waiting time and physician downtime, in order to converge with the optimal appointment length for each class. Bentayeb et al. [14] developed a new appointment scheduler based on a time-of-service prediction model, which is developed using the data mining method. They use classification and regression trees to predict service times with 84% accuracy. They then simulate different scheduling rules to obtain a better sequence of patients. To the best of our knowledge, there are no research articles addressing variable appointment intervals that use an optimization approach for optimal patient assignment.

On the other hand, systems that take into account heterogeneous no-show probabilities usually follow a stochastic programming approach in terms of the randomness of arrivals and service times. This means that, regardless of the appointment interval (fixed or variable), the service time is assumed to follow a certain probability distribution. These models are computationally intensive, which means that instead of using the probabilities directly, the appointment is normally split according to no-show probabilities. For example, Ratcliffe et al. [15] builds a dynamic stochastic scheduler that maximizes profits by controlling two classes of patients with different show rhythms. They develop analytical bounds and approximations that lead to partially optimal scheduling rules. Muthraman and Lawley [16] create a sequential scheduling model with exponential service times and multiple patient no-show probabilities, yet the appointment interval is constant. Zacarias et al. [10] study the analytical properties of accounting for different class probabilities and different appointment intervals in the scheduling of a full day. For example, they conclude that in the presence of homogeneous probabilities and variable appointment times, the patient should be scheduled according to the rule of the shortest processing time first (SPT). Yan et al. [17] develop a model for scheduling sequential appointments considering patient choice and service fairness simultaneously. They use stochastic programming that uses distinct groups of patients grouped by no-show probabilities and homogeneous appointment intervals. Samorani and Harris [18] determine the impact of the probabilistic classifier in scheduling appointments with no-shows. They try several classifiers to obtain N classes of patients in terms of their probabilities of no-shows. They then use a stochastic mixed-integer scheduler with random arrivals and service time and appointment interval determinants and constants.

An alternative idea to the use of stochastic optimization could be to predict the no-show rates and assume deterministic arrivals and service times. The recent availability of Electronic Health Records (EHR) and advances in data science has made it possible to improve this wide variety of scheduling systems. This is because modern predictive techniques applied to EHRs are capable of estimating the probability of patient no-show, which can be used to improve the scheduling system [4]. Regarding deterministic systems, Savelsbergh and Smilowitz [19] are the first to define the probabilities of no-shows for six different categories of patients depending on their preferences (strong or weak) for three different time windows (AM, noon, or PM). These environmental conditions were integrated into an online linear integer program to optimize patient allocation. Later on, Ruiz Hernández et al. [11] proposed a mixed deterministic integer program. The model is probabilistic in the sense that it incorporates the expected income of the center weighted by the probabilities of no-show predicted for each patient. This was the first model to incorporate no-show rates, rather than using an N class approach to obtain different classes of patients in terms of no-show. The present paper proposes an offline scheduling system that extends Ruiz Hernández's work by including the variable appointment interval required for each patient. As it will be seen in the experiments, the inclusion of this information allows to improve considerably the performance of the system.

The contributions of this paper are the following: (1) the inclusion of further heterogeneous probabilities that consider information's about the patient, day and time of the appointment, month, and the indirect waiting time (lead time); (2) the inclusion of the variable appointment interval in a linear binary deterministic problem for an online scheduling system; (3) the development of a model for a weekly scheduling system with dynamic prioritization and differentiation for new patients that maximizes the expected revenue of the center and indirectly minimizes the doctor's idle time; (4) the application of the model to a health center in Madrid that potentially mitigates the effects of patient no-shows.

## 3. The Probabilistic Patient Scheduling Problem with Time Variable Slots

In this section, the mathematical formulation of the proposed patient scheduling model is presented. As discussed above, it takes into account the patients' no-show probabilities and the consultation times required by each patient. The goal of the model is to maximize the center's expected revenue through the reduction of no-shows. The model distinguishes between two types of patients (first visits and show-up visits). In addition, it takes into account the time the patient has been waiting for an appointment to assign a priority parameter that is updated every week. It also takes into account some policy requirements that set the minimum proportion of first visits that have to be scheduled each week.

Before describing the model, the notation that will be used is presented:

Sets:

*I*: days of the week;

*T*: time slots in any given day;

*K*: set of patients to be scheduled for an appointment during the reference week.

Parameters:

*q*: proportion of the number of available slots that must be allocated to first visits;

*d*_*k*_: binary parameter indicating if a patient *k* ∈ *K* has high (*d*_*k*_ = 0) o low (*d*_*k*_ = 1) priority;

*Z*_*k*_: binary parameter indicating if a patient *k* ∈ *K* is a first visit (*Z*_*k*_ = 1) or follow-up (*Z*_*k*_ = 0).

*P*_*itk*_: probability that patient *k* ∈ *K* will show-up to an appointment in {*i*, *t*}, for all *i* ∈ *I* and *t* ∈ *T*;

*w*_*z*_: revenue obtained either from a first visit (*z* = 1) or follow-up (*z* = 0).

*t*_*k*_: number of time slots required by the patient in their consultation.

*h*_1_: slack parameter for the minimum number of slots that can be allocated in one day.

*h*_2_: slack parameter for the maximum number of slots that can be allocated in one day.

Variables:

*x*_*itk*_: binary variable that takes the value 1 if the patient *k* ∈ *K* is assigned to slot {*i*, *t*}, for all *i* ∈ *I* and *t* ∈ *T*;

*x*_*k*_^*T*^: binary variable that takes the value 1 if the patient *k* ∈ *K* is referred back to the waiting list.

With this notation, taking into account that the operator ⌈·⌉ denotes the ceiling function (minimum integer not below), the model is formulated as follows:

(1) $$\begin{array}{c} \max\;\underset{i\in I}{\sum }\underset{t\in T}{\sum }\underset{k\in K}{\sum }x_{itk}P_{itk}\left(Z_{k}w_{1}+\left(1-Z_{k}\right)w_{0}\right), \end{array}$$

(2) $$\begin{array}{c} s.t\underset{k\in K\;}{\sum }\underset{t\in T\;|\;\tilde{t}\geq t>\tilde{t}-t_{k}}{\sum }x_{itk}\leq 1,\forall i\in I,t\in T, \end{array}$$

(3) $$\begin{array}{c} \underset{i\in I}{\sum }\underset{t\in T}{\sum }x_{itk}+x_{k}^{T}=1,\forall k\in K, \end{array}$$

(4) $$\begin{array}{c} \underset{\text{i}\in \text{I}}{\sum }\underset{t\in T}{\sum }\underset{k\in K}{\sum }x_{itk}t_{k}Z_{k}\geq b_{4}, \end{array}$$

(5) $$\begin{array}{c} \underset{\text{i}\in \text{I}}{\sum }\underset{t\in T}{\sum }\underset{k\in K}{\sum }x_{itk}t_{k}\left(1-d_{k}\right)\geq b_{5}, \end{array}$$

(6) $$\begin{array}{c} \underset{k\in K\;}{\sum }\underset{t\in T\;|\;\tilde{t}\geq t>\tilde{t}-t_{k}}{\sum }x_{itk}\geq \underset{k\in K\;}{\sum }\underset{t\in T\;|\;\tilde{t}+1\geq t>\tilde{t}+1-t_{k}}{\sum }x_{itk},\forall i\in I,t\in T\backslash \left|T\right|, \end{array}$$

(7) $$\begin{array}{c} \underset{k\in K}{\sum }\underset{t\in T}{\sum }x_{itk}t_{k}\geq \left|T\right|+h_{1},\forall i\in I, \end{array}$$

(8) $$\begin{array}{c} \underset{k\in K}{\sum }\underset{t\in T}{\sum }x_{itk}t_{k}\leq \left|T\right|+h_{2},\forall i\in I, \end{array}$$

(9) $$\begin{array}{c} x_{itk},x_{k}^{T}\in \left\{0,1\right\},\;\forall i\in I,t\in T,k\in K, \end{array}$$

where

(10) $$\begin{array}{c} b_{4}=\min\left\{\underset{k\in K}{\sum }Z_{k}t_{k},\left\lceil q\left|I\right|\left|T\right|\right\rceil \right\},\;b_{5}=\min\left\{\underset{k\in K}{\sum }\left(1-d_{k}\right)t_{k},\left|I\right|\left|T\right|-b_{4}\right\} \end{array}$$

The objective function maximizes the clinic's expected revenue. Note that when *w*_0_ = *w*_1_ = *w*, the objective function maximizes the expected show-up rate; that is, it maximizes the weighted show-up rate. The set of constraints (2) ensures that only one patient is seen at a time. The constraints (3) guarantee that if the patient does not schedule in the reference week, they are sent back to the waiting list. As we are working with binary variables, it is also ensured that each patient is not scheduled more than once in a week. Constraint (4) ensures at least the minimum time is used for new patients (first visits). Constraint (5) grants that low priority patients are not scheduled until all high priority patients have been scheduled. Constraints (6) force the next slots of the day to be empty if one slot is. This ensures that either all slots are filled continuously or the rest of the day's slots remain empty. Finally, constraints (7) force the time spent in a day to be within acceptable limits.

It should be noted that this model is an extension of the probabilistic model developed in. That study proposed a model to maximize the expected revenues based on no-show probabilities. It considered the distinction between new (first visits) and old patients and imposed priority for patients with long waiting times. However, the model did not take into account scheduling different appointment times, which can help to attend more patients in a week. Mathematically, this difference is seen in a change from the unit of time of appointment to a 5-minute slot. Moreover, the meaning of assigning a slot to the patient, *k* ∈ *K*, changes. In this case, it means that the patient is programmed to enter the appointment in that time slot, while the subsequent *t*_*k*_ − 1 slots must all be equal to zero (see equation (2)). Constraints (4) and (5), which are weighted by the time the patient spends in an appointment, also change. Another contribution of our model is that it forces the assigner not to leave empty slots with the set of constraints (6). Finally, as in our proposal, doctor's working time is not restricted to the number of appointments; constraints are added (7) to ensure that the time limits are not exceeded.

## 4. The Scheduling Process

The scheduling process in the reference health facility used in this study, and for which the model is proposed, works as follows:

1. A waiting list is available with the patient's information for the appointment, including the number of weeks on the waiting list (sojourn), whether the patient is a first (new) visit or not, and the patient's consultation time. New patients are added to the list at the time the appointment is requested and the sojourn is initialized at one
2. The list of patients (referred to as a buffer) to be passed to the scheduler each week is constructed as follows:

- The system first selects the patients with the longest waiting time (sojourn) and assigns them high priority (*d*_*k*_ = 0). This group contains both first visits (*Z*_*k*_ = 1) and follow-up visits (*Z*_*k*_ = 0)
- If the legal minimum number of slots dedicated to follow-up patients has not been filled ( ⌈(1 − *q*) |*I*||*T*|⌉), the system sequentially adds patients in decreasing order of sojourn until the previous condition is met (or the waiting list is left empty). In all but the last iteration, patients are assigned high priority (*d*_*k*_ = 0). This group contains both first visits (*Z*_*k*_ = 1) and follow-up visits (*Z*_*k*_ = 0)
- Finally, if the number of first visits in the buffer is below the legal requirements (⌈*q* |*I*||*T*|⌉), the system sequentially adds first visits in decreasing order of sojourn until the legal requirements are met or there are no first visits left to include. These patients have low priority (*d*_*k*_ = 1) and are first visits (*Z*_*k*_ = 1).

(3) After the buffer is selected, the system passes the lists of candidates to be scheduled to the probabilistic model with variable time (1). Once the appointment schedule is obtained, the patients who did not receive an appointment are sent back to the waiting list with their original sojourn values

## 5. Numerical Experiments

In order to evaluate the performance of our model, an experiment has been conducted that reproduces the routine of the psychiatric department of the Fundación Jiménez Díaz hospital in Madrid.

### 5.1. Probabilities Estimation

To estimate the probabilities of no-show for each patient, we used a database with 76,658 appointments belonging to 5261 patients. The average no-show rate on the dataset is 14.05%. Each appointment was described by 97 predictors commonly used to predict no-shows [1]. This set of predictors contained demographic variables, a set of variables that characterize the patient's previous attendance behavior, variables about the patient's condition, and variables related to the appointment. A logistic regression model with L1 regularization was used to obtain the no-show probabilities. This model, commonly known as Lasso Regression, has been previously used to predict no-shows because of its ability to automatically select variables and because of its interpretability [20]. The variables included in the model contain the day of the week, time, and lead time, which allowed to obtain specific and differentiated probabilities for each patient, day of the week, month, time, and sojourn value.

### 5.2. Experimental Setup

We now describe the procedure used to reproduce the scheduling process during a week in the reference center (presented in Section 3). For an illustration of this process, see Figure 1: flow chart of the experimental setup.

The experiment simulates 48 weeks of a doctor attending patients for six hours from Monday to Friday. These hours are equivalent to 72 slots of 5 minutes each day for a total of 360 slots to be covered throughout the week. Therefore, it is assumed that the doctor does not use extra slots (parameter *h*_2_ = 0). Each appointment lasts between 20 and 30 minutes, which means that each patient requires between 4 and 6 slots per consultation. Consequently, each week, the doctor attends between 60 and 90 patients with an average of 75 if the probabilistic model with variable time proposed is adopted.

The experiment assumes that the center has a list of patients where those who have been waiting for the longest have waited 8 weeks. This list is generated at random. The simulation is performed as follows:

- At the beginning of each week, a set of patients (℘) is generated who ask for an appointment. This is done by generating a random number according to a discrete uniform distribution in [62, 66]. This number is used to randomly select patients from the database so that the proportion of first visits is respected. The selected patients are added to the end of the waiting list with a sojourn value of one. These patients are common to all the scheduling approaches. In the case of model with variable time slots, we assume that times follow a discrete uniform distribution in [4, 6].
- As described above, the buffer of patients to be passed to the scheduler is obtained from the waiting list
- The probabilistic model with variable time (1) assigns the day and time of the appointment to different patients in the buffer. Those patients not assigned return to the waiting list
- Attendance is simulated for each patient, based on their estimated show-up probabilities. If a patient attends the appointment, the center obtains the corresponding profit (70 € per new patient, 50 € per follow-up), and the patient is removed from the waiting list. Otherwise, the patient can request an appointment again with a probability of 0.3, denoted by *p*_*r*_, or leave the waiting list definitively with a probability of 0.7. If the patient reschedules, they are returned to the waiting list with a sojourn value of zero. At the end of the week, the sojourn value of all patients is increased by one

Parameter values are summarized in Table 2. It is important to point out that these values have been provided by the health center basis for this study. In this way, simulation experiments reproduce the expected performance of the center if the proposed system was implemented during an entire year.

### 5.3. Results

We now present the results obtained in the experiment. The performance of the proposed model is compared with the following: (i) the system currently implemented in the health center which assigns the patient to the first available slot with a fixed duration of 30 minutes (FIFO constant); (ii) the system which would assign each patient to the first available slot but would use the estimate of the number of slots they would need (FIFO variable); and (iii) the model proposed by Ruiz-Hernandez et al. [11] that assigns patients based on their probabilities using patient constant appointment time (Time constant). Our model will be referred to as time variable. All models are coded with CPLEX Solver for mathematical optimization in MATLAB R2020a, and the experiments have been conducted in a PC with an Intel Core I9 (2.6-4.5) GHz and 32 GB RAM processor.

Table 3 shows the average results of the simulation over the 48 weeks, including computing times of the different methods. As can be seen, the proposed model achieves better results in terms of the number of patients in the queue and indirect waiting times. Similarly, the center's profit and the doctor's idle time are increased and reduced, respectively, with this approach. These results are achieved while keeping no-show rates at acceptable levels, just behind those of the time constant scheduling model. With respect to the computing time, our model exceeds the time required for existing methods. Nonetheless, the total computing time for allocating all the patients in a week (~32 seconds) is perfectly assumable for an offline scheduling system.

For a more graphic assessment of the results, the cumulated performance measures over the course of each week are presented.  Figure 2(a) shows the number of people on the waiting list for each week. In constant time models, since no more than 60 appointments can be assigned per week, the number of people on the waiting list increases over time. On the other hand, if we compare the variable time models, we can see that the probabilistic model presents better results, by making an assignment that minimizes the effects of the no-shows. It is important to note that the proposed model does not manage to keep the waiting list steady. This is due to the fact that the number of patients is too small in relation to the number that can be assigned. This could be solved either by increasing the number of patients arriving each week or by reducing the center's operating times.

Figure 2(b) shows the sojourn value, i.e., the average number of weeks a patient has to wait before being scheduled for an appointment. As in the previous graph, in constant time systems, the average waiting time for patients increases over the weeks. This is a consequence of not having enough capacity to assign all patients. In contrast, the variable FIFO model remains stable over time but fails to reduce the sojourn value throughout the simulation. Finally, the probabilistic model with variable time not only decreases the time but takes it to the minimum values.

Figure 2(c) shows the cumulated profits. Probabilistic models have higher benefits than the rest. Of these, the model with variable time obtains better revenues, since under this approach, a greater number of patients can be seen and their attendance probability is maximized.

Figure 2(d) shows the cumulated doctor's inactivity time. It should be noted that the constraint added in the probabilistic model ensures that no slots can be left empty throughout the day unless subsequent appointments are not scheduled, see (7). The same applies to the FIFO model. This means that the inactive time of the doctors is highly associated with the number of no-shows. The other factor with direct impact in the doctor inactive time is the difference between the deterministic service time and the scheduled time, which directly affects constant-time models. As in the previous graph, variable time systems offer better results, as they take into account the real patient service times. Among them, the proposed model has a lower cumulative doctor inactive time.

The same pattern can be seen in Figure 2(e), which shows the number of cumulated no-shows. The models with variable time present fewer no-shows, and within them, the model with constant time presents less cumulated no-shows.

Finally, Figure 2(f) presents the complementary of the previous graphic, that is, the number of assigned patients who showed up. Again, models with variable time present better indicators over time since they can allocate a larger number of patients.

## 6. Conclusions

In this article, we have addressed the problem of no-shows in health centers. This problem causes significant damage to the centers, ranging from increased waiting times for patients to severe financial losses. To solve this problem, we have proposed a scheduling system based on a probabilistic scheduling with variable time model together with dynamic priority allocation scheme. The system is based on the solution of a mixed-integer programming model that maximizes the expected profits of the clinic, differentiating between first and follow-up visits. The model minimizes the impact of no-shows on the expected revenues based on the patient's show probabilities and their appointment time.

The model is based on individual estimates of patients' show appointment probabilities. These probabilities have been estimated by using a logistic regression model with L1 regularization (lasso), because of its ability to select variables automatically. In addition, the model can handle different patient appointment times. These values have been simulated based on information provided by the health center from which the data were extracted.

The experiments show that while both the waiting list and the waiting times are increased in the models with constant time, the proposed model is able to reduce the waiting list by 30% and the waiting times by 50% with respect to their values at the beginning of the simulation. The proposed model is also capable of increasing the cumulated earnings by more than 50%, while reducing the cumulated doctor's idle time by more than 40%, with respect to the current system used at the health center.

There are several opportunities for future research. The first is to extend the probabilistic model with variable time developed to allow overbooking. Similarly, the model could be extended to more environmental factors affecting scheduling such as walk-in, early cancelations, and patient preferences. Finally, appointment times could be estimated, just as the attendance probabilities, in order to obtain more realistic results.

To conclude, the proposed model is capable of working in a way that minimizes the probability of a patient missing an appointment, while allowing for more patients to be seen. It has proven to dramatically outperform models with constant time, as well as the variable time extension of the current hospital system.

## Figures and Tables

**Figure 1:** Flow chart of the experimental setup.

**Figure 2:** Weekly simulation results.

**Table 1:** Comparison across recent studies.

Study	Modeling approach	No-shows	Service time	App. interval	Scheduling	
Cayirli et al. [12] (2006)	Rules	1-class	Long\short (deterministic)	Variable	Online
Huang and Verduzco [13] (2015)	Rules	1-class	Objective (deterministic)	Variable	Online
Bentayeb et al. [14] (2019)	Rules	1-class	Predicted (deterministic)	Variable	Online
Ratcliffe et al. [15] (2012)	SP (analytical)	2-class (simulated)	Fixed	Fixed	Offline
Muthraman and Lawley [16] (2008)	SP (analytical)	N-class (simulated)	Exponential (stochastic)	Fixed	Online
Zacarias et al. [10] (2014)	SP (analytical)	N-class (simulated)	Log-normal (stochastic)	Fixed	Online
C. Yan et al. [17] (2015)	SP	N-class (simulated)	Exponential (stochastic)	Fixed	Online
Samorani and Harris [18] (2019)	SMIP	N-class (predicted)	Fixed	Fixed	Online
Savelsbergh and Smilowitz [19] (2016)	ILP	N-class	Fixed	Fixed	Offline
Ruiz Hernández et al. [11] (2019)	MIP	Predicted Probabilities	Fixed	Fixed	Offline
*Proposed scheduling*	*ILP*	*Predicted Probabilities*	*Variable*	*Variable*	*Offline*

**Table 2:** Parameter of the simulation.

Parameters	Values
*q*	0.3
*w*_1_	70
*w*_0_	50
*h*_1_	3
*h*_2_	0
∣*I*∣	5
∣*T*∣	72
*p*_*r*_	0.3
*t*_*k*_	*U*[4, 6]
∣℘∣	*U*[62, 66]

**Table 3:** Average weekly simulation results.

	FIFO constant	FIFO variable	Time constant	Time variable
Patient in the queue	688.449	532.918	672.979	356.143
Average sojourn value (weeks)	9.951	7.787	9.824	5.089
Center's profit	2703.673	3199.184	3434.286	4130.612
Doctor inactive time (minutes)	484.695	210.920	417.145	154.695
No-show rate	0.124	0.120	0.081	0.085
Computing time (seconds)	0	0.002	17.554	32.332

## Data Availability

Answer: No. Comment: The data used to support the findings of this study were supplied by the Jimenez Díaz Hospital under license and so cannot be made freely available. Requests for access to these data should be made to Enrique Baca-García.
